This article has been retracted.

# lncRNA HOTTIP Recruits EZH2 to Inhibit PTEN Expression and Participates in IM Resistance in Chronic Myeloid Leukemia

**DOI:** 10.1155/2022/9993393

**Published:** 2022-09-08

**Authors:** Jing Liu, Lin Yang, Xiaojun Liu, Lu Liu, Menghan Liu, Xuefeng Feng, Jianmin Luo

**Affiliations:** Key Laboratory of Hematology, Second Hospital of Hebei Medical University, Shijiazhuang 050000, China

## Abstract

**Objective:**

To investigate that HOTTIP suppressed PTEN gene expression and was involved in IM resistance in chronic myeloid leukemia through recruitment of EZH2 protein.

**Methods:**

Seventy-one cases of bone marrow monocytes diagnosed with CML in the Second Hospital of Hebei Medical University from 2018 to 2021 were selected. These patients were diagnosed with CML by bone marrow morphology, immunology, molecular biology, and cytogenetics, of which 36 were sensitive to IM and 35 were resistant to IM. We selected K562 and IR-K562 cells preserved in the laboratory as our subjects to study the expression levels of HOTTIP in the bone marrow cells of IM CML-resistant patients and IM-resistant cells.

**Results:**

In this study, we found that HOTTIP was highly expressed in the bone marrow and cell lines of CML patients resistant to Imatinib mesylate (IM). In in vitro experiments, lentiviral knockdown of HOTTIP inhibited CML cell proliferation and promoted apoptosis, and knockdown of HOTTIP also increased sensitivity to IM. Mechanistically, highly expressed HOTTIP is involved in the biological process of IM resistance by recruiting Zeste homologous protein 2 enhancer (EZH2) to inhibit the expression of phosphatase and Tensin homologous protein (PTEN) genes.

**Conclusions:**

We confirmed that HOTTIP and EZH2 are highly expressed in IM-resistant patients and IM-resistant CML cell lines. In CML cell lines, HOTTIP is involved in regulating the proliferation and apoptosis of CML cells and resistance to IM.

## 1. Introduction

Chronic myeloid leukemia (CML) is one of the major types of leukemia, accounting for 15% of adult leukemias, with a global annual incidence of approximately 1.6 to 2/100,000 [1]. Chronic granulocytic leukemia has no clear etiology, but its development is closely related to characteristic abnormalities of the pH chromosome [2]. The clinical presentation of patients is associated with progression [3]. The main features of chronic granulocytic leukemia are elevated peripheral blood granulocytes, anemia, basophilia, and infantile cellularity, usually accompanied by features such as splenomegaly and thrombocytosis, mainly due to a clonal disease occurring in pluripotent hematopoietic stem cells [4]. In addition, Chinese patients with CML are younger than those in Western countries. Epidemiological surveys in several regions of China have shown that the median age of CML onset is 45-50 years, whereas the median age of CML onset in Western countries is 67 years [1]. CML is the first human tumor that has been shown to be associated with chromosomal abnormalities, as patients have translocated chromosomes 9 and 22, forming a new BCR-ABL fusion gene. This fusion gene expresses a unique 210 kDa tyrosine phosphoprotein kinase (p210BCR-ABL) [5]. Before the advent of tyrosine kinase inhibitors (TKI), the efficacy of conventional chemotherapy was unsatisfactory, the conditions for bone marrow transplantation were demanding, and patient prognosis was poor, with a 10-year survival rate of less than 20% [6]. In 2001, the first TKI drug was approved and marketed internationally, indicating that CML treatment entered the era of targeted therapy. Since then, the prognosis of patients has greatly improved, with the 10-year survival rate increasing to 85-90% [7]. Currently, most CML patients can benefit from TKI drug therapy, and some patients can even achieve treatment-free remission (TFR), but about 10% of patients still experience drug resistance or disease progression, and acquired drug resistance has become a major challenge for CML treatment [8].

In the mammalian genome, less than 2% of transcripts have protein-coding functions, and the remaining 98% are noncoding RNAs (ncRNAs). Based on the length of nucleotide sequences, ncRNAs can be classified into short-stranded ncRNAs (sncRNAs) and long-stranded ncRNAs (lncRNAs) [9]. HOTTIP is a 4,665 bp long lncRNA transcribed from the distal end of the human HOX gene and plays an oncogenic role in various human solid tumors [10]. The exosomal lncRNA HOTTIP can enhance the expression of karyopherin subunit *α*3 by binding miRNA-214 and is involved in mitomycin resistance in colon cancer [11]. HOTTIP predicts low survival in gastric cancer and promotes B-cell lymphoma 2 (BCL-2) expression by binding miRNA-216a-5p, thereby reducing autophagy-related death and promoting cisplatin resistance in gastric cancer cells [12]. In hematologic tumors, HOTTIP is highly expressed in acute myeloid leukemia (AML) cell lines and AML-M5 patients, which is associated with survival rates. In AML cell lines, the combination of HOTTIP and miRNA-608 can upregulate the expression of DDA1 and thus promote the proliferation of AML cells [13]. However, whether HOTTIP can play a role in CML remains to be investigated.

Abnormal epigenetic modifications play an important role in tumor formation and progression, and it is currently one of the hot targets for antitumor drugs [14]. Epigenetics refers to the regulation of transcriptional activation or repression of genes without altering the DNA sequence [15]. Many drugs targeting epigenetic modifications have been used clinically (e.g., azacitidine for myelodysplastic syndromes and vorinostat for cutaneous T-cell lymphoma) with good clinical results [16]. Epigenetic disorders include DNA methylation, histone modifications, chromosome remodeling, and RNA interference, which can be involved in the pathogenesis of CML [17]. Histone lysine methyltransferase enhancer of zeste homolog 2 (EZH2), the core catalytic subunit of comb repressive complex 2 (PRC2), can trimethylate the lysine 27 (K27) site of histone H3 (H3K27me3), i.e., with no change in total histone, the expression level of H3K27me3 increases, and the methylated histones bind more tightly to DNA, inhibit DNA binding to transcription factors, silence oncogenes, and promote tumorigenesis [18]. EZH2 is highly expressed or gain-of-function mutated in many tumor cells, and these changes are closely associated with poor patient prognosis [19]. Meanwhile, EZH2 is required to maintain the function of many cancer stem cells, such as breast cancer, pancreatic cancer, glioma, and acute myelogenous leukemia [20–22]. Recent studies have shown that EZH2 knockdown can inhibit the self-renewal and survival of leukemia stem cells (LSCs) and increase the sensitivity of LSCs to IM [23].

In the present experiments, we investigated the expression and interaction of HOTTIP, EZH2, and PTEN genes in CML cells. We confirmed that HOTTIP and EZH2 were highly expressed in IM-resistant patients and IM-resistant CML cell lines. Highly expressed HOTTIP repressed the transcription of PTEN gene and downregulated its expression by recruiting EZH2, thereby activating the downstream signaling pathway of PTEN and promoting the proliferation of CML cells. In CML cell lines, HOTTIP is involved in regulating the proliferation and apoptosis of CML cells and resistance to IM.

## 2. Materials and Methods

### 2.1. General Information

Seventy-one cases of bone marrow mononuclear cells diagnosed with CML at the Second Hospital of Hebei Medical University from 2018 to 2021 were selected. These patients were diagnosed with CML by bone marrow morphology, immunology, molecular biology, and cytogenetics. Among them, 36 cases were sensitive to IM, and 35 cases were resistant to IM. Details of the patients are shown in Table 1, and bone marrow mononuclear cells from 40 healthy individuals were selected as a control group. Patients with vital organ dysfunction, pregnant women, and those who did not provide informed consent were excluded. The ethics committee of the Second Hospital of Hebei Medical University approved the experiment, and all patients' families signed the informed consent form.

### 2.2. Cell Culture and Transfection Method

We selected K562 and IR-K562 cells preserved in the laboratory as our research subjects. The K562 cells were cultured using an RPMI 1640 medium (Gibco); the IR-K562 cells were cultured using a Dulbecco's medium (IMDM). The RPMI 1640 and IMDM mediums were supplemented with 10% FBS and 100 *μ*g/mL penicillin and streptomycin, respectively. Cells were incubated at 37°C in an incubator saturated with 95% air and 5% carbon dioxide (Thermo, Waltham, MA, USA).

A lentiviral vector containing short hairpin sh-HOTTIP and sh-EZH2 or overexpressing HOTTIP was constructed (synthesized by Shanghai Jikai Gene Company). First, the cells were inoculated with a complete culture medium to prepare cells with a density of 1 × 10^5^, and then the infection enhancer was added. Then, the virus volume was calculated according to the MOI value of 30 for the k562 and IR-K562 cells (which refers to the ratio of virus particles and cell numbers that were used when 80% of cells were infected) and transfected into the cells. After 48 h of infection, infection efficiency was observed by fluorescence, and the stably transfected cells were screened with a final concentration of 2 *μ*g/mL puromycin.

### 2.3. Cell Viability Assay

We used a CCK-8 reagent to detect cell viability. The cells of different treatment groups with a cell count of 1 × 10^5^ were counted and spread into 96-well plates. After 48 h of treatment, 10 *μ*L of CCK-8 reagent was added into each well. After the 96-well plates were put into a 37°C incubator for reaction for a period of time, the OD value at 450 nm was detected.

### 2.4. Cell Apoptosis Assay

The Annexin V/FITC/PI apoptosis kit (BD Biosciences, Franklin, New Jersey, USA) was used to detect apoptosis. The cells of different treatment groups with a cell count of 5 × 10^5^ were spread in a 24-well plate. After the cells were treated separately for 48 h, they were collected and washed twice by PBS and placed into a flow tube. After being diluted with the kit, the buffer was resuspended and collected into the flow tube. Each tube was labeled with 5 *μ*L of APC and 10 *μ*L of the PI antibody. After standing in the dark for 10 min, the apoptotic cells were detected by Beckman Coulter. Data analysis (Beckman Coulter) was performed using the Kaluza software.

### 2.5. Flow Cell Cycle

Cell cycle detection was performed using a DNA content detection kit (Yisheng Biology, 40301ES50) with a cell count of 1 × 10^5^ for the single cell suspension preparation. After the cells were precipitated by centrifugation at 1,000 g for 5 min, the supernatant was discarded. The cells were rinsed once with 1 mL of precooled PBS, mixed gently with 1 mL of precooled 70% ethanol, and fixed at 4°C for more than 2 h or overnight. The precipitated cells were centrifuged and resuspended in precooled PBS. 10 *μ*L of propidium iodide stock solution and 10 *μ*L of RNase A solution were added to 0.5 mL of staining buffer and the mix. Each cell sample was added with 0.5 mL of the prepared propidium iodide staining solution, and the cells were gently mixed and resuspended. After incubation in the dark for 30 min at 37°C, flow cytometry analysis (Beckman, FC500) was performed.

### 2.6. Colony-Forming Assay

The hemicellulose-based semisolid culture medium was configured by dissolving 2 g methylcellulose powder into 50 mL ultrapure water, which was then shaken and mixed evenly and subjected to high-pressure sterilization. Once the temperature was reduced to 37°C after sterilization, 50 mL RIPM 1640 with two times concentration was added, and the mixture was repeatedly cooled and shaken until no clots were found. The samples were separately packaged and stored at −20°C. The cells were resuspended using a culture with 20% FBS, and the cell density was adjusted to 2 × 10^3^/mL. The cells were added into a methyl cellulose semisolid culture medium with the same volume and mixed evenly by shaking. One milliliter of the mixed suspension was sucked and placed into a 35 mm Petri dish. Three Petri dishes were repeated and kept in a cell incubator with 5% CO2 at 37°C. After the culture sat in a cell incubator with saturated humidity for 20 days, the number of colonies that had more than 50 cells were counted under a microscope.

### 2.7. RNA Extraction and Quantitative Real-Time PCR

Centrifuged bone marrow mononuclear cells were collected, RNA was extracted by using a TRIzol (Invitrogen, Carlsbad, CA, USA) reagent, RNA concentration was calculated, cDNA was extracted by using a reversal kit (Funeng, Guangzhou, China), a real-time quantitative polymerase chain reaction (PCR) was subsequently carried out using an all-in-one kit (Funeng, Guangzhou, China), Tm was synthesized according to the primers, and the annealing temperature and the cycle number of each gene to be amplified were determined to be 95°C for 15 s, 60°C for 30 s, and 72°C for 20 s when 40 cycles were carried out after the preexperiment. The real-time PCR results were analyzed using *β*-actin as the internal reference. The primer sequence for the target gene was as follows: HOTTIP forward primer 5′-TGAGAACATTCATGCGG-3′; reverse primer 5′-GAATGCAATCCAAAGCCTTC-3′; EZH2 forward primer 5′-GACCTCTGTCTTACTTGTGGAGC-3′; reverse primer 5′-CGTCAGATGGTGCCAGCAATAG-3′; PTEN forward primer 5′-ACCAGGAC-CAGAGGAAACCT-3′; reverse primer 5′-GCTAGCCTCTGGATTTGACG-3′; GAPDH forward primer 5′-GCAAATTCCATGGCACCGTC-3′; and reverse primer 5′-TCGCCCCACTTGATTTTGG-3′.

### 2.8. Western Blot Analysis

After the cells were washed with PBS and collected, we extracted the protein using RIPA and determined the protein concentration using the BCA protein concentration kit (Boster Biological Company, Ltd., Wuhan, China). According to the instructions, the proteins were separated by 10% and 6% SDS-PAGE gels, transferred to the PVDF membrane by electrophoresis, blocked by TBST containing 5% defatted milk powder for 1 h, and incubated overnight at 4°C with the following primary antibodies: EZH2 (1 : 600, Boster Biological Company, Ltd., Wuhan, China), PTEN (1 : 600, Boster Biological Company, Ltd., Wuhan, China), BCL-2 (1 : 600, Boster Biological Company, Ltd., Wuhan, China), BAX (1 : 600, Boster Biological Company, Ltd., Wuhan, China), cleaved caspase-3 (1 : 600, Boster Biological Company, Ltd., Wuhan, China), H3 (1 : 600, Boster Biological Company, Ltd., Wuhan, China), H3K27me3 (ab192985, Abcam, CA, USA), and GAPDH (1 : 8,000; Abways Technology, New York, NY, USA; AB0035). After sitting overnight, the TBST was shaken and washed for 10 min three times. The PVDF membrane was incubated with a goat anti-rabbit secondary antibody (1 : 10,000, Boster Biological Company, Ltd., Wuhan, China) for 1 h by shaking, and protein imaging and gray value analysis were performed using the ImageJ software (UVP, LLC, Upland, CA, USA) after the activation signal of the ECL luminescent agent was used.

### 2.9. Fluorescence In Situ Hybridization (FISH)

A clone vector for amplification was prepared to obtain an antisense strand probe. IR-K562 cells were passaged and washed with PBS and then spread into 24-well plates. Cell climbing plates were placed into each well and fixed with 4% paraformaldehyde for 10 min. Cells were permeabilized with 0.5% Triton X-100 for 10 min. The digestion was stopped by adding a 100 mm glycine solution. 100 *μ*L of a hybridization buffer was added into each well. Then, 200 *μ*L of 1× DAPI staining solution were added, and gelatin sealing tablets were added dropwise onto the glass slides. The slides were taken out, and the cells were reversed toward the slide. Observation and photographing were conducted under a laser confocal microscope (Nikon Eclipse Ti, Tokyo, Japan).

### 2.10. RIP-qPCR

RNA binding to the EZH2 protein was obtained by RIP in IR-K562 cells and verified by qPCR for the target lncRNA. The cells were collected, resuspended in a complete lysis buffer equal to the volume of the cells, blown, and mixed. The IP group samples were set to be negative control IgG, and the experimental group was set to be EZh2. 100 *μ*L of RIP Wash Buffer and 5 g of antibodies (EZH2 antibody 21800-1-AP, ProteinTech) were added to each IP group. RNA for input and IP groups were extracted using the TRIzol reagent. The purified RNA was analyzed for samples using a RT-qPCR.

### 2.11. Animal Experiment

Sixteen male nude mice (16–20 g, 5–6 weeks of age) with severe combined immunodeficiency were purchased (SPF Biotechnology Company, Ltd., Beijing, China). All mice were raised at an ambient temperature of 18–22°C and a relative humidity of 50–60%. Lentivirus was used to stably knock down HOTTIP IR-K562 cells, and negative control cells were injected subcutaneously into the left dorsal side of each mouse (0.5 × 10^6^ cells per injection). Tumor size, volume, and body weight were dynamically observed. On day 25, sh-con and sh-HOTTIP were, respectively, divided into two groups, the control group and the Tazemetostat group, and 250 mg/kg BID was given by gavage for 18 days. The tumor-bearing mice were sacrificed for sample collection and detection. The research animal experiments were approved by Hebei Provincial Animal Experimental Committee and conducted in accordance with their guidelines.

### 2.12. Detection of EZH2 Enzyme Activity

Follow the steps in the EZH2 activity colorimetric assay kit. First, the standard curve was prepared using the methylated standard substance known in the kit, and the relationship was plotted with OD value as the *Y* axis and standard substance concentration as the *X* axis. Then, according to the slope, the absolute number generated in the sample could be determined.

### 2.13. Target Prediction

Prediction of the HOTTIP and EZH2 binding regions was performed using RPISeq (http://pridb.gdcb.iastate.edu/RPISeq/) and catRAPID (http://service.tartaglialab.com/page/catrapid_group).

### 2.14. Statistical Analysis

The SPSS22.0 statistical software was used for data analysis, and the mean ± standard deviation ($\bar{x}\pm SD$) was used for measurement data. *t*-test was used for comparison of means between two groups, and paired *t*-test was used for comparison of means before and after intervention in the same group. The *χ*^2^ test was used for comparison of rates *p*<0.05 was considered a statistically significant difference.

## 3. Results

### 3.1. lncRNA HOTTIP Is Highly Expressed in Imatinib-Resistant Patients and Imatinib-Resistant Cell

Previous studies have confirmed that HOTTIP is highly expressed in the bone marrow cells of some solid tumors and in AML patients, but the expression level of HOTTIP in CML patients and cell lines is still unknown. In this study, RT-qPCR confirmed the expression of HOTTIP in the bone marrow cells of IM-resistant patients was higher than that of IM-sensitive patients (Figure 1(a)). In the cell line IR-K562, cells showed significantly higher IC50 (6.35 ± 0.31 *μ*mol/L) of IM than K562 cells (0.37 ± 0.03 *μ*mol/L); after 48 h of IM treatment, the apoptotic rate of K562 cells (65.36 ± 5.25%) was significantly higher than that of IR-K562 cells (7.74 ± 2.44%). The results above confirmed that IR-K562 cells were highly resistant to IM (Figures 1(b) and 1(c)), which proved that IR-K562 cells were IM-resistant cell lines, and the expression of HOTTIP in IR-K562 cells was superior to that in K562 cells (Figure 1(d)). The above results confirmed HOTTIP was highly expressed in the bone marrow cells of IM CML-resistant patients and IM-resistant cells.

### 3.2. Lentivirus Knocks Down HOTTIP in IR-K562 Cells, Inhibits Cell Proliferation, Blocks Cells in G1 Phase, and Promotes Apoptosis

To elucidate the biological function of HOTTIP in CML resistance to IM, we used IR-k562 cells as the research object and lentivirus to stably transfect sh-con and sh-HOTTIP. We found that the lentivirus transfected sh-HOTTIP successfully and knocked down the expression of HOTTIP in CML cells (Figure 2(a)), and we observed the functional changes of CML cells after knocking down HOTTIP. We found that the cell viability (as determined by CCK) after knocking down the HOTTIP group and the colony-forming ability (as determined by the clone formation experiment) of the sh-HOTTIP group were lower than those of sh-con (all *p* values < 0.05) (Figures 2(b) and 2(c)), and compared with sh-con, the cells were blocked in G1 phase (as determined by flow cytometry) (Figure 2(d)), and the apoptosis after knocking down the HOTTIP was higher than that of sh-con (as determined by flow cytometry) (Figure 2(e)). After knocking down HOTTIP, the antiapoptotic protein BCL-2 was decreased, and the apoptotic proteins BAX and c-caspase were increased (Figure 2(f)). The above results confirmed the lentivirus stably inhibited the proliferation of CML cells and promoted the apoptosis of CML cells after knocking down the HOTTIP.

### 3.3. Overexpression of HOTTIP Reduced the Sensitivity of K562 Cells to IM

In the first part of our study, it was proved that the expression of HOTTIP in IM-sensitive K562 cells was lower than that in drug-resistant IR-K562 cells. Therefore, we constructed a lentivirus overexpressing HOTTIP and transfected K562 cells to observe how the sensitivity to IM changed after the cells overexpressed HOTTIP. First, observe the lentivirus transfection efficiency. The FITC-positive labeled cells were the cells successfully transfected. As shown in Figure 3(a), the cells successfully transfected in K562 cells accounted for 93% of all cells. The efficiency of lentiviral was further validated using RT-qPCR, which indicated that the lentivirus successfully overexpressed HOTTIP expression levels compared to controls (Figure 3(a)).

Further, we analyzed how the cell sensitivity to IM changed after overexpression of HOTTIP in K562 cells. First, K562 cells were divided into the control group (lv-con) and HOTTIP overexpression group (lv-HOTTIP). The inhibitory efficiency of IM on these two cells was tested by CCK-8, and the results showed that the IC50 (0.93 ± 0.6 *μ*mol/L) of lv-HOTTIP cells against IM was higher than that of lv-con cells (0.60 ± 0.04 *μ*mol/L, *P* <0.05). The difference was statistically significant (Figure 3(b)). In terms of apoptosis, the cells in the two groups were treated with DMSO or 0.5 *μ*mol/L IM for 48 hours, and the cells were divided into the lv-con group, the lv-con+IM group, the lv-HOTTIP group, and the lv-HOTTIP+IM group. The results showed that after the cells were stimulated with the same concentration of IM, the apoptosis rate in the lv-HOTTIP+IM group (10.46 ± 0.96%) was lower than that in the lv-con+IM group (28.96 ± 1.25%), and the difference was statistically significant (Figure 3(c)). The expression of apoptosis-related proteins was detected by Western blot, and the results showed that after the cells were stimulated with the same concentration of IM, compared with the lv-con+IM group, the expression of antiapoptotic protein BCL-2 in the lv-HOTTIP+IM group was increased, and the expression of apoptotic proteins BAX and c-caspase-3 was decreased (Figure 3(d)). The above results demonstrated that overexpression of HOTTIP in IM-sensitive K562 cells decreased the sensitivity to IM, and overexpression of HOTTIP induced drug resistance in K562 cells.

### 3.4. Knocking Down HOTTIP Increases the Sensitivity of IR-K562 Cells to IM

The above studies have confirmed that overexpression of HOTTIP can reduce the sensitivity of K562 cells to IM. Next, we investigated how cells respond to IM after knocking down the expression of HOTTIP in IR-K562 cells that are resistant to IM. First, the lentivirus transfection efficiency was observed. The FITC-positive labeled cells were the cells successfully transfected. As shown in the figure, the cells successfully transfected into IR-K562 cells accounted for 94.1% of all cells. The efficiency of lentivirus knockdown was further verified by RT-qPCR, which indicated that lentiviruses successfully knocked down the expression level of HOTTIP in IR-K562 cells when compared with the control group (Figure 4(a)).

To further analyze how IR-K562 cell sensitivity to IM changes after the HOTTIP is knocked down, first, IR-K562 cells were divided into the control group (sh-con) and the HOTTIP knockdown group (sh-HOTTIP). The inhibitory efficiency of IM on these two cells was tested by CCK-8, and the results showed that the IC50 (4.32 ± 0.31 *μ*mol/L) of sh-HOTTIP cells against IM was lower than that of sh-con cells (5.95 ± 0.58 *μ*mol/L), *p* < 0.05, and the difference was statistically significant (Figure 4(b)). In terms of apoptosis, the cells of the two groups were treated with DMSO or 3 *μ*mol/L IM for 48 hours, which were divided into the sh-con group, the sh-con+IM group, the sh-HOTTIP group, and the sh-HOTTIP+IM group. The results showed that after the cells were stimulated with the same concentration of IM, the apoptosis rate in the sh-HOTTIP+IM group was 45.86 ± 5.91% higher than that in the sh-con+IM group 17.9 ± 2.92%, and the difference was statistically significant (Figure 4(c)). Western blot was used to detect the expression changes of apoptosis-related proteins, and the results showed that after the cells were stimulated with the same concentration of IM, compared with the sh-con+IM group, the expression of antiapoptotic protein BCL-2 in the sh-HOTTIP+IM group was decreased, and the expressions of apoptotic protein BAX and c-caspase-3 were increased (Figure 4(d)). The above results demonstrate that knocking down HOTTIP in IR-K562 cells resistant to IM increases cell susceptibility to IM.

### 3.5. HOTTIP Recruits EZH2 to Inhibit PTEN Expression and Participates in IM Resistance

To clarify which pathway HOTTIP is involved in the process of IM resistance in CML cells, we used the bioinformatics website to predict the regulatory genes. The binding score of HOTTIP and EZH2 predicted by RPIseq was 0.75, and the binding region of HOTTIP and EZH2 predicted by catRAPID ended up being selected for preliminary verification (Figure 5(a)). We confirmed the subcellular localization of EZH2 and HOTTIP in IR-K562 by FISH and found that there was an overlapping localization area of EZH2 and HOTTIP in the nucleus (Figure 5(b)). In addition, RIP and RT-qPCR experiments confirmed whether EZH2 and HOTTIP were bound to each other (Figure 5(c)). The results suggest HOTTIP was highly expressed in the RNA-protein complex to which the EZH2 antibody was bound, proving that EZH2 and HOTTIP are bound to each other. After the lentivirus knocked down HOTTIP in IR-K562 cells, RT-qPCR and Western blot results showed that both mRNA and the protein levels of EZH2 decreased, and HOTTIP regulates EZH2 expression (Figure 5(d)).

Studies have shown that the expression of PTEN increases after the knockdown of EZH2 in various solid tumors. Therefore, we have verified whether the expression of PTEN is changed after the inhibition of EZH2 in CML cells. To determine the expression level of EZH2 in CML patients and cell lines, we conducted verification in CML patients and CML cell lines. Results of RT-qPCR and WB verification indicated the expression levels of EZH2 mRNA and protein in bone marrow cells of CML IM-resistant patients were higher than those of IM-sensitive patients and healthy donors. Similarly, the expression levels of EZH2 mRNA and protein in the IM-resistant cell line IR-K562 were higher than those in K562 cells (Figure 5(e)), proving EZH2 might also be involved in IM resistance. Constructed EZH2-knockdown lentivirus to transfect IR-K562 cells, the mRNA and protein expressions of EZH2 and PTEN were detected by RT-qPCR and Western blot. With the decrease of EZH2 expression, the expression of H3K27me3 protein was decreased, and the expression of PTEN mRNA and protein was increased (Figure 5(f)), suggesting that EZH2 could regulate the expression of PTEN gene.

In our previous work, it was confirmed that HOTTIP was involved in CML's resistance to IM, and RIP experiment confirmed that HOTTIP combined with EZH2. To further verify that HOTTIP was involved in CML's resistance to IM through EZH2, we knocked down HOTTIP and EZH2 simultaneously from IR-K562 and then observed the changes of cell function. IR-K562 cells were divided into three groups, a control group (sh-con), a group in which the HOTTIP was depressed (sh-HOTTIP), and a group in which the HOTTIP and EZH2 were both depressed (sh-HOTTIP+sh-EZH2). First, the proliferation and apoptosis were detected by CCK-8 method and flow cytometry. The results showed that compared with the sh-HOTTIP group, the sh-HOTTIP+sh-EZH2 group exhibited further decreased cell proliferation and further increased apoptosis (with 3 *μ*mol/L IM stimulation) (Figures 6(a) and 6(b)). When the three groups of cells were treated with IM at the same concentration, the sh-HOTTIP+sh-EZH2 group had a decreased IC50 for IM as compared with the sh-HOTTIP group (Figure 6(c)). Compared with the sh-HOTTIP group, the expressions of EZH2 and methylated H3 (H3K27me3) in the sh-HOTTIP+sh-EZH2 group were further decreased, and the expressions of PTEN were further increased. When treated with 3 *μ*mol/L IM, the expressions of BCL-2 in the sh-HOTTIP+sh-EZH2 group were further decreased, and the expressions of c-caspase-3 were further increased. These results confirmed that HOTTIP was involved in Imatinib resistance by regulating EZH2 to inhibit PTEN expression in CML cells (Figure 6(d)).

### 3.6. HOTTIP Inhibits PTEN Expression In Vivo

Tazemetostat is a “first-in-class” EZH2 inhibitor developed by the FDA and marketed for the treatment of inoperable, metastatic, or locally advanced epithelial sarcoma [24] (Figure 7(a)). To verify whether Tazemetostat is effective in reducing EZH2 activity, we treated IR-k562 cells with different concentrations of Tazemetostat, and ELISA results showed that with increasing concentrations of Tazemetostat, the activity of EZH2 enzyme gradually decreased, the expression of H3K27me3 protein decreased, and PTEN protein Tazemetostat successfully inhibited the activity of EZH2 enzyme and promoted the expression of PTEN protein (Figure 7(b)).

IR-K562 cells transfected with sh-con and sh-HOTTIP were used for tumorigenesis in nude mice. After tumorigenesis, tumor size and weight changes were dynamically observed and measured in tumor-bearing mice. Tumor size was recorded at days 5, 10, 15, 20, and 25, and the results showed that the tumor volume in the HOTTIP knockdown group was significantly smaller than that in the control group (Figure 7(c)). At day 25, we used Tazemetostat to interfere with the EZH2 enzyme activity. The sh-con and sh-HOTTIP were divided into two groups, control (normal saline) and Tazemetostat 250 mg/kg (BID) by gavage for 18 days. Tumor-bearing mice were sacrificed, and then samples were collected and tested. The results showed that the tumor volume was significantly reduced in the Tazemetostat group after knockdown of HOTTIP compared with the normal saline group, and the difference was statistically significant (*p* < 0.05) (Figure 7(c)). Meanwhile, WB and immunohistochemical experiments confirmed that the expression levels of PTEN and c-caspase3 were higher in the Tazemetostat group than in the normal saline group (Figures 7(d) and 7(e)). The above results confirmed that HOTTIP knockdown could inhibit the growth of nude mouse xenografts, while PTEN expression was further increased after Tazemetostat was used to interfere with EZH2 enzyme activity, suggesting that HOTTIP regulates EZH2 in vivo to inhibit PTEN expression.

## 4. Discussion

CML is a myeloproliferative disease in which a fusion gene BCR-ABL, encoding the BCR-ABL tyrosine kinase protein, is formed through molecular biological changes [25]. The first generation TKI Imatinib was invented as a countermeasure. Although most CML patients respond to Imatinib treatment, some patients still fail and relapse due to resistance to IM, and ultimately, the complex and multifactorial biological process leading to clonal changes in the gene is an important cause of targeted drug therapy failure [26]. TKI resistance in CML patients can be divided into BCR-ABL-dependent and BCR-ABL-independent mechanisms, including BCR-ABL mutations and overexpression, abnormal drug transporter activity, aberrant activation of compensatory signaling pathways, DNA repair and genomic instability, epigenetic dysfunction, durability of LSCs, and immune system dysfunction [27]. The understanding of resistance mechanisms has facilitated the advancement of second- and third-generation TKI drugs designed to overcome and suppress BCR-ABL1 mutations. However, despite the advent of next-generation TKI, there are still mutations, such as the T315I mutation, that remain resistant to multiple TKI [28].

There is growing evidence that lncRNAs are associated with tumorigenesis and may serve as prognostic biomarkers in various cancers [29]. HOTTIP is a lncRNA transcribed from the 5′ end of the HOXA gene. Studies have confirmed that HOTTIP is involved in metastasis and progression of several tumors and is associated with prognosis. In hematological tumors, HOTTIP is involved in the pathogenesis of AML and is associated with survival. HOTTIP is aberrantly activated in AML to alter HOXA-driven topology-associated domain (TAD) and gene expression. Deletion of HOTTIP impairs leukemia development in transplanted mice, whereas reactivation of HOTTIP restores leukemic TAD, transcription, and CTCF boundaries that enhanced leukemic progression in AML cells [30]. In this study, we found that HOTTIP was highly expressed in CML patients and that HOTTIP expression was higher in CML patients and IM-resistant CML cell lines than that in patients and IM-sensitive cell lines. In addition, the sensitivity of cells to Imatinib was altered by changing the expression level of HOTTIP, suggesting that HOTTIP plays an oncogene role in CML and is involved in IM resistance.

In the last decade, we have made great progress in studying epigenetic disorders of hematologic neoplasms [31]. EZH2 is the catalytic core component of PRC2 that silences gene expression through trimethylation of H3K27. EZH2 dysregulation and hypertumorigenicity have been observed in a variety of cancers. EZH2 mutations frequently occur in myeloproliferative/myeloproliferative neoplasms, myelodysplastic syndromes, and myelofibrosis, while CML cases are mainly characterized by EZH2 overexpression [18]. Our study showed that EZH2 was highly expressed in bone marrow mononuclear cells from IM-resistant patients.

In CML, high expression of EZH2 was associated with the activation of BCR-ABL, and EZH2 expression was promoted through the STAT5 signaling pathway, which decreased after treatment of CML stem cells with TKI [32, 33]. As a therapeutic target, EZH2 can be used as an adjuvant agent in CML aimed at eliminating residual LSC. Studies have confirmed that the combination of EZH2 inhibitors and TKI can delay leukemia progression, extend survival time in mice, and reduce the disease burden of LSC in in vivo and in vitro experiments [23]. Tazemetostat is a potent and highly selective EZH2 inhibitor with sustained safe anticancer effects in in vitro and in vivo models of mutant B-cell non-Hodgkin's lymphoma, INI1-negative malignant rhabdomyosarcoma, and SMARCA4-negative malignant ovarian rhabdomyosarcoma, and phase 2 clinical studies with Tazemetostat monotherapy in adult B-cell non-Hodgkin's lymphoma are ongoing [24]. In our study, the activity of EZH2 decreased after Tazemetostat treatment of CML cells. As the concentration of Tazemetostat increased, the expression of PTEN protein increased, indicating that Tazemetostat inhibited the expression of EZH2 and thus promoted the expression of PTEN gene. Since Tazemetostat is able to suppress tumors, further studies are needed to determine whether combining targeted EZH2 inhibition with TKI has a synergistic effect and exerts a stronger antitumor effect.

In in vivo experiments, after tumor formation in nude mice, the tumor volume and weight in the HOTTIP group were lower than those in the control group, suggesting that the HOTTIP knockout group could inhibit the growth of transplanted tumors in vivo. After tumor formation in nude mice, normal saline and Tazemetostat treatment further interfered with the activity of EZH2. Tazemetostat reduced the expression of H3K27me3 and promoted the expression of PTEN gene in vivo, thus exerting an effect on drug-resistant cells.

In this study, we demonstrated that HOTTIP is highly expressed in the bone marrow of IM-resistant patients and that HOTTIP inhibits PTEN gene expression by recruiting EZH2 protein. HOTTIP recruits EZH2 to participate in drug resistance, suggesting that Tazemetostat could be used as an adjuvant in CML patients with high HOTTIP expression. However, whether the EZH2 inhibitor Tazemetostat can be used in the clinic remains to be validated in future animal models and clinical trials.

## Figures and Tables

**Figure 1:** HOTTIP is highly expressed in CML. (a) RT-qPCR was used to detect. Note: HOTTIP level in BM-MNCs of CML patients and BM-MNCs of healthy donors. Normalized to GAPDH. ^∗∗∗^*p* < 0.001 vs. NC. (b) K562 and IR-K562 cells were treated Imatinib in different concentrations for 48 h. Imatinib IC50 was evaluated by CCK-8 assay. ^∗∗∗^*p* < 0.001. (c) Cell apoptosis rate was detected by flow cytometry using Annexin V-APC/PI staining. The right panel shows the apoptosis rate from three independent experiments. ^∗∗^*p* < 0.01 vs. sh-con. (d) RT-qPCR was used to detect HOTTIP levels in CML cell lines (K562 and IR-K562).

**Figure 2:** (a) IR-K562 was transfected with specific sh-RNA of HOTTIP or negative. Note: sh-RNA (sh-con). RT-qPCR was used to detect HOTTIP level. (b) IR-K562 was transfected with specific sh-RNA of HOTTIP or negative sh-RNA (sh-con). CCK-8 analysis was used to detect cell proliferation. (c) CML cells were prepared as (a), and cell proliferation was detected by colony formation assay. ^∗∗^*p* < 0.01 vs. sh-con. (d) CML cells were prepared as (a), and cell apoptosis rate was detected by flow cytometry using Annexin V-APC/PI staining. The right panel shows the apoptosis rate from three independent experiments. ^∗^*p* < 0.05, ^∗∗^*p* < 0.01 vs. sh-con. (e) Western blotting for protein levels in IR-K562 cells transfected with sh-HOTTIP and sh-con.

**Figure 3:** Upregulation of HOTTIP decreases the sensitive of IM in K562 cells. Note: (a) K562 was transfected with specific lv-RNA of HOTTIP or negative lv-RNA (lv-con). RT-qPCR was used to detect HOTTIP level. (b) K562 cells were transfected with specific lv-HOTTIP or negative lv-con and treated with different Imatinib concentrations for 48 h. CCK-8 analysis was used to detect cell inhibition. ^∗∗^*p* < 0.05 vs. sh-con. (c) K562 cells were transfected with specific lv-HOTTIP or negative lv-con and treated with Imatinib for 48 h. Cell apoptosis was detected by flow cytometry using Annexin V/APC/PI. The right panel shows the apoptosis rate from three independent experiments. ^∗∗^*p* < 0.01 vs. sh-on. (d) Western blotting for protein levels in K562 cells transfected with lv-HOTTIP or negative lv-con and treated with IM (0.5 *μ*M) or DMSO for 48 h.

**Figure 4:** Knocking down HOTTIP increases the sensitivity of IR-K562 cells to IM. Note: (a) IR-K562 was transfected with specific sh-RNA of HOTTIP or negative sh-RNA (sh-con). RT-qPCR was used to detect HOTTIP level. CCK-8 analysis was used to detect cell proliferation. (b) IR-K562 cells were transfected with specific sh-HOTTIP or negative sh-con and treated with different Imatinib concentrations for 48 h. CCK-8 analysis was used to detect cell inhibition. ^∗^*p* < 0.05 vs. sh-con. (c) IR-K562 cells were transfected with specific sh-HOTTIP or negative sh-con and treated with different concentrations of Imatinib for 48 h. Cell apoptosis was detected by flow cytometry using Annexin V/APC/PI. The right panel shows the apoptosis rate from three independent experiments. ^∗∗^*p* < 0.01 vs.sh-on. (d) Western blotting for protein levels in IR-K562 cells transfected with sh-HOTTIP or negative sh-con and treated with IM (3 *μ*M) or DMSO for 48 h.

**Figure 5:** HOTTIP regulates EZH2 to inhibit PTEN expression. Note: (a) catRAPID predicted binding region of HOTTIP and EZH2. (b) FISH analyzed the localization of EZH2 and HOTTIP in IR-K562 cells. (c) RIP-PCR were used to test the interaction between EZH2 and HOTTIP. ^∗^*p* < 0.05 vs. IgG. (d) RT-qPCR and Western blot were used to measure EZH2 mRNA and protein level after knocking down HOTTIP. (e) Western blot analysis was used to measure EZH2 in BM-MNCs of CML patients. Right panel, bar chart of protein densitometric analysis. ^∗∗∗^*p* < 0.001. RT-qPCR was used to detect EZH2 level in BM-MNCs of CML patients. Normalized to GAPDH. ^∗∗∗^*p* < 0.001 vs. NC. Western blot analysis was used to measure EZH2 protein level in IR-K562 and K562 cells. Right panel, bar chart of protein densitometric analysis. ^∗∗∗^*p* < 0.001; RT-qPCR was used to detect EZH2 mRNA level in CML cell lines (K562 and IR-K562). Normalized to GAPDH. ^∗∗∗^*P* < 0.001 vs. NC. (f) RT-qPCR and Western blot were used to detect EZH2 and PTEN mRNA and protein levels after transfecting with specific sh-con or sh-EZH2. ^∗∗∗^*P* < 0.001 vs. DMSO.

**Figure 6:** HOTTIP work through EZH2 to participate in drug resistance. Note: (a) IR-K562 cells were transfected with specific sh-HOTTIP or both sh-HOTTIP+sh-EZH2. The CCK-8 analysis was used to detect cell proliferation. (b) Cell apoptosis was detected by flow cytometry using Annexin V/APC/PI. The right panel shows the apoptosis rate from three independent experiments. (c) IR-K562 cells were prepared with different Imatinib concentrations for 48 h. The CCK-8 analysis was used to detect cell inhibition. (d) WB was used to detect protein levels.

**Figure 7:** The effect of HOTTIP on CML cell in vivo. Note: (a) Tazemetostat drug structure. (b) Analysis of H3K27me3. PTEN expression in IR-K562 cells treated by Tazemetostat with different concentrations for 48 h. ^∗∗∗^*p* < 0.001 vs. DMSO. (c) IR-K562 cells were engineered to stably knock down HOTTIP, and the cells were then subcutaneously injected into the nude mice to establish CML xenograft tumors. Tumor volumes were monitored by direct measurement. ^∗^*p* < 0.05, ^∗∗^*p* < 0.01, and ^∗∗∗^*P* < 0.001 vs.sh-con. Representative tumor sizes of xenograft mice in each group. The xenograft tumor wet weight in each group of mice. ^∗^*p* < 0.05, ^∗∗^*P* < 0.01 vs. sh-con. (d) Immunohistochemistry stain was used to measure the PTEN, c-caspase3 protein levels in xenograft tumors. (e) Western blot was used to detect the H3K27me3, PTEN, and c-caspase3 protein levels in xenograft tumors.

**Table 1:** Characteristics of CML patients included in the study.

Characteristic	Sensitive (*n* = 36)	Resistance (*n* = 35)
Age (years)	57.36±10.58	51.29±15.49
Male/female (*n*/*n*)	24/12	20/15
WBC count, 109/L	258 (54-426)	185 (69-553)
Haemoglobin level (g/L)	82.86±32.99	74.08±28.56
Platelet count, 109/L	164±23.74	251±40.14

## Data Availability

The simulation experiment data used to support the findings of this study are available from the corresponding author upon request.
